# Which Occupations Did People Engage in during Lockdown? A European Cross-Sectional Descriptive Survey by Generation

**DOI:** 10.1155/2023/3979298

**Published:** 2023-08-21

**Authors:** Cynthia Engels, Lauriane Segaux, Amandine Ibanez, Florence Canouï-Poitrine, Charlotte Lafont

**Affiliations:** ^1^Univ Paris Est Creteil, INSERM, IMRB, CEpiA Team, F-94010 Creteil, France; ^2^Faculty of Health, Univ Paris Est Creteil, F-94010 Creteil, France; ^3^AP-HP, Henri Mondor Hospital, Public Health Service, F-94010 Creteil, France

## Abstract

**Objective:**

The primary objective was to describe the occupations people engaged in more frequently during lockdown than before the coronavirus disease 2019 pandemic as a function of generation. The secondary objectives were to (i) describe the levels of importance, performance, and satisfaction for these occupations and (ii) identify factors affecting the levels of importance, performance, and satisfaction.

**Method:**

We conducted an online, cross-sectional survey of young adults (YAs, aged 18-39), middle-aged adults (MAs, aged 40-59), and older adults (OAs, aged 60 or over).

**Results:**

2534 participants (YAs: 47%, MAs: 33%, and OAs: 20%) cited 4500 occupations. The occupations in which people most engaged were leisure occupations (67%), followed by productive occupations (31%) and then self-care (2%) occupations. YAs gave a median (interquartile range) importance score of 8 (6; 9) to leisure, 8 (7; 10) to productivity, and 8 (7; 10) to self-care. MAs gave a median importance score of 8 (6; 10) to leisure, 8 (7; 10) to productivity, and 8 (7; 10) to self-care. OAs gave a median importance score of 8 (7; 10) to leisure, 8 (7; 9) to productivity, and 9 (8; 10) to self-care. In a pre-/postlockdown comparison, the changes in performance scores among YAs were +5 (3; 6) for leisure, +4 (2; 5) for productivity, and +4 (3; 6) for self-care. Among MAs, these changes were, respectively, +4 (3; 6), +3 (2; 5), and +4.5 (3; 6). Among OAs, these changes were, respectively, +3 (1; 5) for leisure, +3 (2; 5) for productivity, and +2 (0; 4) for self-care. The changes in satisfaction scores among YAs were +3 (0; 5) for leisure, +3 (0; 5) for productivity, and +3 (1; 6) for self-care. Among MAs, these changes were, respectively, +3 (0; 5), +2 (0; 4), and +5 (0; 6). Among OAs, these changes were, respectively, +2 (0; 4), +2 (0; 4), and +2 (0; 4).

**Conclusions:**

Lockdown led to stronger engagements in quiet leisure and alternative forms of socialization. Occupational therapists may have a role in helping community-dwelling people to balance and structure their new daily routine.

## 1. Introduction

The 2020 pandemic of coronavirus disease 2019 (COVID-19, caused by severe acute respiratory syndrome coronavirus 2 (SARS-CoV-2) and that could be spread through small liquid droplets in the breath [1]) prompted many countries to go into lockdown (i.e., “mandatory mass quarantine” [2]) for varying periods. In France, for example, trips outside the home were restricted to an hour and a radius of 1 km unless the person could justify a “compelling reason.” People outside the home had to carry identification and a time-stamped declaration. Much the same system was applied in Italy. In Spain, outdoor sports were prohibited [3–5]. According to the World Federation of Occupational Therapists (WFOT) [6], “populations around the world have been required to adjust and make compensations to usual routines in order to participate in ongoing or newly acquired occupations that are necessary for daily life.” To study the impact of those global changes from an occupational perspective, we conducted occupational participation during the COVID-19 lockdown in Europe during spring 2020, by Generation (COPACO) study. Occupational disruption has been defined as “a state that is usually temporary or transient rather than prolonged” [7]. Furthermore, occupational disruption “occurs when a person's normal pattern of occupational engagement is disrupted due to significant life events (such as having a baby), environmental changes (such as moving house or location), becoming ill or sustaining an injury from which full recovery is expected” [7]. During the COVID-19 pandemic in spring 2020, the risk of occupational disruption affected the general population and not just “disabled people and others marginalized and disempowered by poverty, racism and the legacies of colonialism” [8]. However, “from our clients and the research evidence, we [occupational therapists] know that resilience in face of crisis is the norm rather than the exception” [8].

The Canadian Model of Occupational Performance and Engagement (CMOP-E) [9] describes three occupational domains (self-care, leisure, and productivity), each of which has three subgroups (i.e., personal care, functional mobility, and community management for self-care; quiet recreation, active recreation, and socialization for leisure occupations; and paid/unpaid work, household management, and play/school for productive occupations). The CMOP-E shows how the interactions between a person's affective, cognitive, physical, and spiritual characteristics; their physical, institutional, cultural, and social environment; and their occupations can lead to occupational engagement or occupational disruptions. Hence, the ability to engage in other occupations and the nature of these occupations can vary as a function of several variables. For example, a range of studies have shown that the nature of engaged occupations can change with age [10, 11]. We therefore wondered whether people of different ages manage differently during lockdown. In the first publication, we explored occupational disruption during lockdown, by generation [12]. In the present study, we sought to determine how opportunities for occupational engagement were taken up during lockdown, in order to objectify and quantify occupations that were more frequently performed by the general population in a context of environmental restrictions that had never been applied before on such a broad scale. Consequently, the study's primary objective was to describe the occupations that were more frequently engaged in during lockdown than in the prepandemic period, as a function of the generation. The secondary objectives were to (i) describe the levels of importance, performance, and satisfaction for these occupations (again, as a function of the generation) and (ii) explore factors possibly affecting the levels of importance, performance, and satisfaction for these occupations.

## 2. Materials and Methods

### 2.1. Study Design and Participants

We performed an online, cross-sectional survey of adults (aged 18 and over) locked down in their homes (i.e., not in institutions) in the European Union (EU) and Switzerland. In early April 2020, the world's 15 most affected countries included nine European countries: Spain, Italy, Germany, France, the United Kingdom, Switzerland, Belgium, the Netherlands, and Austria [13]. These countries were therefore among the first to implement national disease containment measures, including lockdown (Deutsche [14]). In view of the EU's common legislation and regulatory framework, the present study focused on the 28 EU member states at that time and the nonmember Switzerland, which is surrounded by EU member states. We assumed that people living in institutions were already subject to occupational restrictions on a regular basis and so excluded this population from the study.

### 2.2. Study Instrument

We created a 32-question online questionnaire based on the literature data in general [15, 16] and the CMOP-E in particular [9]. The first part of the questionnaire addressed the person's characteristics via six multiple-choice questions. The second part addressed the person's physical and social environment via seven multiple-choice questions. As we wanted to offer survey participants an opportunity to include specific, person-centred occupations, we used an open tool that was consistent with our theoretical framework. Hence, the third part of the questionnaire was based on the Canadian Occupational Performance Measure (COPM) [17]. Participants were asked to state up to three occupations in which they had engaged more frequently during lockdown. Next, on a 1-to-10 numerical scale, the participant rated each occupation's self-perceived importance (i.e., “how important is it for you to perform…?”), performance (i.e., “how successful are you when you…?”), and satisfaction (i.e., “how satisfied are you with the way you …?”) during the prepandemic period and during lockdown. An additional question addressed the frequency of the occupation during the prepandemic period and during lockdown, on a seven-point scale ranging from “every day” to “never.” The last part of the questionnaire (seven questions, not analyzed here) addressed interactions and feelings during lockdown, as well as an open question for comments. The French version of the survey was initially tested on five adults. We then had the questionnaire translated into the main official languages of the nine European countries most affected by COVID-19 in April 2020 (Dutch, English, French, German, Italian, and Spanish). Each questionnaire was tested by a native speaker and then adjusted if necessary. The estimated completion time was around 10 minutes. The questionnaire can be obtained on request from the authors.

### 2.3. Data Collection

The online questionnaire was created using SurveyMonkey with the “anonymous” option to prevent IP addresses from being recorded. A specific link to the questionnaire was generated for each language. To produce snowball sampling, the links were published on various webpages (Institut National de la Santé et de la Recherche Médicale (INSERM), the Clinical Epidemiology and Aging (CEpiA) research group, and the WFOT) and social media (Facebook, Twitter, and LinkedIn) on April 9, 2020, and were removed on May 8, 2020. In line with the EU's legislation on anonymous surveys that do not record personal data, approval of the study by an independent ethics committee was not required. Information about the study was given on the first page of the questionnaire, and consent to participation in the study was inferred through the completion of the questionnaire. The main endpoint was the nature of the occupational domains (leisure, productivity, or self-care) in which occupations were more frequently engaged during lockdown compared with the previous (prepandemic) period. The secondary endpoints were (i) the CMOP-E's occupational subdomains (i.e., quiet recreation, active recreation, or socialization for leisure occupations; household management, paid/unpaid work, or play/school for productive occupations; and personal care, functional mobility, or community management for self-care occupations [17]) in which people engaged more frequently during lockdown than in the previous period and (ii) ratings of importance and changes in satisfaction, performance (on a 10-point Likert scale), and frequency (on a 7-point Likert scale), relative to the previous period.

### 2.4. Analysis

Continuous variables were described as the median (interquartile range (IQR)). Categorical variables were described as the number (percentage). As a generation has typically been defined as people born in the same 20-year period [18], we defined the younger adult (YA) group as comprising people aged between 18 and 39 in 2020, the middle-aged adult (MA) group as comprising people aged 40 to 59, and the older adult (OA) group as comprising people aged 60 or more. After testing the data's normality for the outcome measures, the groups' characteristics were compared by using the Kruskal-Wallis test for continuous variables and Pearson's chi-squared test or Fisher's exact test (as appropriate) for categorical variables. All tests were two-tailed, and the threshold for statistical significance was set to *p* < 0.05. When the overall *p* value for the differences between the three groups was <0.2 for a given domain (i.e., self-care, productivity, or leisure), subdomain (active recreation, quiet recreation, etc.), or sub-subdomain (participating in sports, cultural outings, etc.), we performed pairwise comparisons; the *p* values were corrected using the false discovery rate method. A multivariate logistic regression was used to identify the independent variables associated with more frequently engaged occupations (our dependent variable): the analysis was adjusted for the sex, type of environment (house/flat, urban area/countryside), socioprofessional status (craftsperson/trader/company manager/farmer, executive/intellectual profession, or worker/employee/intermediate profession), and country of residence (France, other countries). The multivariate logistic regression was conducted on an individual level (i.e., an individual could only account for 0 or 1 in the studied variable, even if they could have quoted more than one occupation in the domain of interest). Associations were assessed as the adjusted odds ratio (aOR) and its 95% confidence interval (CI), together with the *p* value in a Wald test. Missing data were not imputed. All statistical analyses were performed with Stata software (version 15.0, StataCorp LLC, College Station, TX, USA).

For qualitative questions, the thematic content was analyzed by the first author with regard to the CMOP-E theoretical framework [9]; each occupation was allocated to one of the three domains and then to the appropriate subdomain and sub-subdomain. Given that the detailed information on occupation domains typically gathered during the COPM interview was not recorded for each respondent, we kept as close as possible to the examples given in Appendix A of the COPM booklet [17]. For example, “cooking” was always allocated to household management, and “intellectual learning” was always allocated to play/school—even though a detailed interview might have given a better understanding of the value that the respondent placed on an occupation. Furthermore, the classification of a given leisure occupation as “active” or “quiet” can depend on the age of the person doing it [10]. Hence, in order to be able to compare age groups, we again referred to the examples given in the COPM booklet.

## 3. Results

A total of 3241 completed questionnaires were received: 165 were excluded because the respondent had not stated their date of birth, and 542 were excluded because the respondent did not answer the question about engagement in occupations. Hence, 2534 completed questionnaires were included in our analysis. The sample came from 20 different European countries. The predominant country was France (*n* = 2190, 78%), where the survey had been launched. The other participants were from Belgium (*n* = 90), Switzerland (*n* = 69), Spain (*n* = 36), Germany (*n* = 28), the United Kingdom (*n* = 27), Austria (*n* = 22), Italy (*n* = 20), Ireland (*n* = 12), Denmark (*n* = 6), the Netherlands (*n* = 6), Portugal (*n* = 5), Greece (*n* = 4), Sweden (*n* = 2), Croatia, Finland, Malta, Poland, Romania, and Slovenia (*n* = 1 each). The country of residence was not reported by 11 participants. Given the poorly balanced sample, we compared respondents living in other countries with a random sample (1 : 1) of respondents living in France.

### 3.1. Characteristics of the Study Population

The demographic characteristics of the study population are summarized in Table 1. There were 1179 respondents (47%) in the YA group, 839 (33%) in the MA group, and 516 (20%) in the OA group. There was female predominance, especially among the YAs. Overall, executive or intellectual professions were the best represented. There were more employees (60.6%) and less intermediate professions (18.1%) in France than in other countries (33.9% and 48.2%, respectively; *p* < 0.001). Most of the YAs were workers or students, while the great majority of MAs were workers, and the great majority of OAs were retired. Half of the YAs had been living in a flat during lockdown, while most of the MAs and OAs had been living in a house. Most of the respondents had been living in an urban area; this was more the case in France (64.5%) than in other countries (54.7%; *p* = 0.01). Ninety-eight percent had been living with the same people during lockdown as during the prepandemic period. The majority of YAs and MAs were working/studying from home, while 73% of the OAs, 16% of the MAs, and 23% of the YAs were not working/studying at all during lockdown. Although the great majority of participants did not lose income during lockdown, a partial, major, or even total loss of income was more frequently reported by the YAs (29%) than by the MAs (24%) and OAs (10%) (*p* < 0.001). A total of 401 (16%) respondents stated they did not engage in any particular occupation more frequently during lockdown. The other respondents reported a total of 4519 occupations that were more frequently engaged in: 24% of the respondents mentioned one occupation, 27% mentioned two, and 33% mentioned three (the maximum allowed on the survey questionnaire). Nineteen of these occupations could not be allocated to a CMOP-E domain, and so 4500 were allocated and analyzed (Table 2). As one individual could quote up to three occupations, the rest of our analysis was based on the occupation unit (*n* = 4500) rather than the individual unit (*n* = 2534).

We found that 666 (15%) of the mentioned occupations were new in that they had not been mentioned by the respondent as having been performed before lockdown: there were 350 new occupations (16% of the total) for YAs, 210 (14%) for MAs, and 106 (12%) for OAs. Younger adults were more likely to engage in new occupations than OAs, who were more likely to engage more in previously practiced occupations. The remaining 3834 occupations (85%) had already been performed before the lockdown, albeit less frequently.

Overall, the occupations that were more frequently engaged in during lockdown than during the prepandemic period were leisure occupations (67%), followed by productive occupations (31%) and then self-care occupations (2%). In the univariate analysis, OAs performed more leisure occupations more frequently and productive occupations less frequently; however, the differences were not statistically significant in a multivariate analysis (Table 3).

### 3.2. Leisure

Leisure covered 67% of the occupations that were more frequently engaged in. All three generations reported a change of +2 points (1; 4) in frequency (on a 7-point Likert scale from “every day” to “never”). The results for the importance, performance, and satisfaction scales with regard to leisure are summarized in Table 4.

Although all three generations highlighted quiet recreation occupations, OAs were less likely to report these occupations once the data had been adjusted for other sociodemographic variables (aOR (95%CI) = 0.64 (0.41-0.99) vs. YAs; *p* = 0.05). Reading was the main quiet occupation, followed by crafts—especially among YAs and OAs. Watching TV/series (notably including online shows/concerts) accounted for 6% of the occupations, with no significant differences between the three generations. Smaller proportions of respondents reported playing board games and listening to or playing music. Online gaming was mentioned by YAs more than MAs and OAs (*p* < 0.001). Greater use of digital technology was reported more by OAs (*p* < 0.001). People living in a house were less likely than people living in a flat to engage in quiet recreation during lockdown (aOR (95%CI) = 0.67 (0.53-0.85)).

Twenty-five percent of the occupations that were more frequently engaged in during lockdown corresponded to active recreation. These were especially physical activities and then gardening (mentioned less by YAs; *p* = 0.004). Playing with children accounted for 1% of the occupations mentioned by YAs and MAs, but none of those mentioned by OAs (*p* = 0.003).

Socialization accounted for 4% of the more frequently practiced occupations and was mentioned more by MAs and OAs than by YAs (*p* = 0.03). This mainly corresponded to developing new kinds of relationships through video calls, spending more time than usual on the phone, and spending more time than usual with family members. Socialization leisure accounted for a significantly greater proportion of MAs' reported occupations, even after adjustment for other sociodemographic variables (aOR (95%CI) = 1.56 (1.03-2.34); *p* = 0.03 vs. YAs).

### 3.3. Productivity

Thirty-one percent of the frequent occupations were productive. Overall, the participants reported a median (IQR) change of +2 points (1; 4) in frequency. The results for the importance, performance, and satisfaction scales with regard to productivity are presented in Table 5.

For each generation, the most frequently mentioned productive occupation was household management (24% of the reported occupations). The second most frequently mentioned productive occupation was paid/unpaid work for MAs and play/school for YAs and OAs. The play/school category included all kinds of intellectual learning activity (e.g., learning a foreign language). After adjusting for other sociodemographic data, people living in France were less likely to report paid/unpaid work occupations in their answers.

The household activities mainly comprised cooking for YAs and Mas and household chores for OAs (*p* < 0.001). The third most frequently mentioned occupation was caring for children (especially homeschooling) for YAs and MAs (*p* < 0.001) and DIY for OAs (*p* = 0.1). A smaller proportion of respondents in each generation also mentioned new ways of shopping for groceries—especially online grocery shopping. After adjustment for other sociodemographic variables, women were more likely than men to report household management as being among their more frequent occupations (aOR (95%CI) = 1.54 (1.18-2.02); *p* = 0.002).

Occupations involving paid work mainly consisted of working online and/or from home and were cited more often by MAs (*p* < 0.001). Respondents who were workers, employees, or from intermediate professions were less likely to report paid occupations in the multivariate analysis (aOR (95%CI) = 0.38 (0.18-0.82)) when compared with craftsmen, traders, company managers, or farmers (*p* = 0.01).

### 3.4. Self-Care

Self-care featured in only 2% of the completed questionnaires and was most frequently mentioned by YAs (*p* = 0.002). Only activities from the personal care subgroup were found. YAs, MAs, and OAs reported changes in the frequency of +2 (1; 4), +1 (1; 2), and +2 (1; 3), respectively (*p* = 0.2). The results for the importance, performance, and satisfaction scales with regard to self-care are summarized in Table 6.

Resting was mentioned more by YAs (*p* = 0.004). Most of the other answers were about taking time to care for one's appearance. After adjustment for other sociodemographic variables, people living in a house were less likely to mention personal care occupations (aOR (95%CI) = 0.43 (0.22-0.85); *p* = 0.02).

## 4. Discussion

We analyzed questionnaire data on 4500 newly performed or more frequently performed occupations submitted by 2534 individuals (YAs: 47%, MAs: 33%, and OAs: 20%) across Europe (mainly France: 78%). Our results showed that YAs were more likely to engage in new occupations than OAs, who were more likely to engage more in previously practiced occupations. Overall, the occupations that were more frequently engaged in during lockdown than during the prepandemic period were leisure occupations (67%), followed by productivity occupations (31%) and then self-care occupations (2%).

### 4.1. Lockdown Allowed the Development of Leisure Occupations

Our results showed that adults of all generations started or developed several leisure activities during lockdown. This finding is in line with (i) Paltrinieri et al.'s report in which 84% of the surveyed citizens in the Italian province of Reggio Emilia started new leisure occupations during lockdown [19] and (ii) Huls et al.'s [20] report that respondents spent 11% more time on leisure. More precisely, quiet recreations (typically those practiced at home) accounted for 38% of the 4500 newly performed or more frequently performed occupations in our study; this was especially true for YAs after adjustment for other sociodemographic variables. Fristedt et al.'s study also highlighted the fact that some OAs spent as much time or even more time in quiet leisure pursuits at home (such as genealogy and playing cards) during lockdown as they did before lockdown [21]. In Belgium, Cruyt et al. found that 97% of leisure activities performed by adults at home were continued during lockdown [22].

Previous studies performed in Europe showed that in the prepandemic period (i.e., before the lockdown), (i) 89% of OAs showed an interest in quiet leisure occupations [11] and (ii) 18% of European adults aged 50 and over engaged in quiet leisure more than once a week (22% in France), vs. 9% for people below the age of 50 (8% in France) [23]. Our univariate analysis showed that reading was the most frequent quiet leisure occupation, which is in line with Paltrinieri et al.'s report that 39% of the surveyed citizens in Reggio Emilia read more than before [19]. In our study, this was especially true among OAs. According to Brown's international data [24], YAs read more books, but MAs and OAs spent more time reading on a regular basis; hence, this trend appeared to be maintained during lockdown. On average, the frequency of reading increased by two points (on a 7-point Likert scale) for all generations. In a study conducted in 2018, 17% of French adults of various ages said they would like to prioritize reading if they had more time [25]. Hence, when people do have more time (because other leisure activities like meeting friends and family have stopped, for example), people from all generations seem to reengage with previously performed, quiet leisure activities in general and reading in particular. In this respect, Cruyt et al. found that during the lockdown, restricted occupations were replaced “with other still comparable activities evoking the same purpose or meaning”.

Even when an occupation was not new during the lockdown, the way of engaging in it may have changed; for example, YAs usually read more outside their homes (mainly in public transport) under prepandemic circumstances [25], while this would have been less possible during lockdown. Cruyt et al.'s results also highlighted that some home occupations continued during lockdown but in a different manner [22].

### 4.2. Lockdown Led to More Traditional Daily Routines among Younger Generations

During the prepandemic period, OAs in Europe were twice as likely to engage in household chores and gardening more than once a week than younger generations were [23]. In our study, household management accounted for 24% of the occupations more frequently engaged; this notably comprised cooking (13% for YAs, 11% for MAs, and 4% for OAs), household chores (5% for YAs, 9% for MAs, and 12% for OAs), and caring for children (3% for YAs, 4% for MAs, and 1% for OAs). Paltrinieri et al. also found cooking to be the most frequent new occupation during lockdown [19]. In our study, gardening also accounted for 7% of more frequently engaged occupations (5% for OAs, 7.5% for MAs, and 8% for OAs), but this proportion was much higher (34%) in Paltrinieri et al.'s study [19]. In our study, these “traditional” occupations were still more prevalent among OAs during lockdown (gardening: *p* = 0.004; house chores: *p* < 0.001) but were increasingly taken up by all generations during lockdown. In a study conducted in Jordan, the participants also reported dedicating more time than usual to household chores, cooking, and housework/parenting [26]. In Belgium, researchers found that 98% of the chores done at home were continued during lockdown [22].

In our study, OAs were less likely to report cooking among their more frequent occupations during lockdown (*p* < 0.001). This might be due to the fact that YAs and MAs were at home on work days, when they would otherwise have eaten in a canteen. In contrast, OAs would probably already have had lunch at home on a regular basis. However, the comments recorded during the survey prompt us to hypothesize that this occupation was also broadly engaged in as a leisure activity; for example, the respondents mentioned baking cakes (notably with children) and homemade bread. This is also in line with the results of Malkawi et al.'s qualitative study in Jordan: cooking was used to occupy time and as a pleasant occupation, rather than just for the preparation of food [26].

Furthermore, the nature of several comments in the survey suggested that although lockdown led to occupational disruption, it also provided an opportunity to “take time for oneself”—especially among YAs, of whom 3% of the more frequent occupations were personal care (resting, taking a bath, etc.). As mentioned above, OAs spent more time doing occupations that they already performed previously, while YAs engaged more in new occupations (including some “traditional” occupations). This finding might guide occupational therapists with regard to the adaptation of previous occupations or engagement in new occupations. Hence, the time freed up by lockdown (e.g., time spent commuting and leisure time usually spent away from the house) appeared to be used for “traditional” occupation by all three generation groups in a similar way.

### 4.3. Socialization

Socialization accounted for 4% of the increased occupations. Even though traditional forms of socialization were restricted, other forms developed. For example, the use of digital technologies accounted for a greater proportion of OAs' more frequent occupations during lockdown (*p* < 0.001). More specifically, video calls accounted for 2% of the occupations mentioned overall (*p* = 0.9). On the same lines, Malkawi et al.'s study [26] mentions other form of socialization during lockdown, such as playing music with neighbours each on their respective balconies. In a study conducted in Sweden, OAs also reported that despite greater restriction in their social contacts, they developed new types of social encounter: discussions with neighbours over a hedge, discussions with (grand)children through the window, social media, and video calls [21]. These activities were especially important because Paltrinieri et al. [19] found that support from family and friends was perceived as being helpful during the lockdown.

In a study carried out in Europe before the pandemic, 37% of the OAs and 52% of the under-35s stated that they saw their friends at least once a week [23]. In a qualitative study of OAs conducted in Sweden at the beginning of the pandemic, some of the participants reported spending most of their time alone at home before lockdown [21]. Lockdown might therefore have lessened generational differences in social contacts. Furthermore, people strengthened their family links during lockdown [27]. This strengthening might explain the greater development of socialization among OAs: given that (i) OAs were presented in the media as being more vulnerable and (ii) all generations had more free time at home than usual, the OA's friends and family might have contacted them more than usual. This is an important finding because 63% of the OAs in a European study thought that “aging well” included being surrounded by their loved ones [23]. It remains to be seen whether the stronger links with OAs will persist once the pandemic is over.

### 4.4. The Influence of Gender and Place of Living

Although our study focused on a generational approach, our multimodal analysis revealed that occupations were influenced by gender and the place of living. Indeed, being a woman was positively associated with productivity and households (a subcategory of productivity) in all three age groups. Källdalen et al. [11] found that among OAs, women had a larger number of household management interests than men did. In another study of adults with an average age of 40, women were more likely to be involved in household chores [28]. Our results indicate that in a context of disaster management such as lockdown, those trends are maintained or even reinforced. A report from the UK highlighted the burden of single mothers with children at home during lockdown [29]. Paltrinieri et al. [19] also found that men engaged in fewer occupations than women did during lockdown. Further research might provide a better understanding of how each gender managed during the lockdown.

Regarding the place of living, living in a house was positively associated with developing quiet recreations, play/school occupations, and personal care. This is in line with the results of González-Bernal et al.'s [30] study of 3261 participants in Spain: private access to an outdoor area was positively associated with occupational balance during lockdown. Older adults who participated in Fristedt et al.'s study [21] also reported that living in the countryside (rather than in an urban area) or in a house (rather than in an apartment) made them feel less at risk of being infected with SARS-CoV-2. Further investigations could usefully highlight the interactions between a person's characteristics, his/her environment, and his/her occupations, as described in the CMOP-E.

### 4.5. Importance, Satisfaction, and Performance during the Lockdown

In our study, each category of occupation was given a similar importance score. We found that some median levels of satisfaction and performance were higher during lockdown than before lockdown: the change ranges from +2 to +5 for the satisfaction score and from +1 to +5 for the performance score (Tables 4–6). In other words, people from all generation groups were more satisfied during the lockdown and felt that they performed better in the occupations mentioned. Although self-care was the least frequently mentioned occupation class, the MAs' satisfaction score was 5 points higher during lockdown than during the prepandemic period; this reflects the extra time they took for self-care during lockdown. Except for the performance score recorded by OAs regarding self-care occupations, all the satisfaction and performance score increased by ≥2 points; this is considered to be a clinically significant difference (M. [17]). Although lockdown led to 6549 restricted occupations in the same sample (mainly leisure activities (83%) and productive activities (16%) [12]), it also allowed more engagement in and greater satisfaction with some occupations. Lastly, we observed a two-point difference between YAs and OAs with regard to the change in the leisure performance score. Hence, our results indicate that relative to OAs, YAs might have experienced a greater increase in their performance of leisure occupations during lockdown vs. the prepandemic period.

### 4.6. Study Strengths and Limitations

Our study had several limitations. Firstly, the sampling via social media limited our ability to extrapolate the results to the general population. Indeed, the proportion of people aged 60 or over was 20% in our survey vs. 27% in the French general population [31]. Moreover, the respondents' social and health-related profiles might not be representative of typical respondents aged 60 and over, who are less likely to be able to access and use the Internet. Therefore, the differences between age groups might have been underestimated. Secondly, despite our efforts to spread the survey to other EU countries, a high proportion of our respondents were living in France. However, that still left 344 respondents from 19 other countries. To adjust for this problem, we carried out multivariate sensitivity analyses by comparing respondents living in France with respondents living in other countries: the only significant differences concerned a few specific occupations (walking, cycling, and “other sports”) and paid work. We also adjusted for the country in our multivariate model; there were no significant differences other than for paid/unpaid work. We therefore decided to pool the data from all countries. Thirdly, the sample was predominantly composed of women (77%). Occupations can differ between genders [9, 11, 32]. In particular, the literature data show that women's engagement in leisure activities is less affected by age and worsening health than men's engagement is [33]. However, all our results were adjusted for gender, which enabled us to interpret our results with regard to the generation.

Fourthly, we followed the COPM process as closely as possible, even though the tool's psychometric proprieties were suited to an interview rather than a survey. For the same reason, we collected less information than is usually gathered in a COPM interview and so had to decide on the allocation of an occupation (rather than discussing it with the respondent). However, the online questionnaire method allowed us to obtain 2534 replies in six different languages in a month, which would not have been possible with interviews.

Fifthly, we translated our questionnaire literally and did not perform any cross-cultural validations. However, the questions that might have been influenced by cultural background were open and so were unlikely to have restricted the respondents' ability to cite their occupations. Sixthly, only one author analyzed the data from the COPM process. However, she relied on the examples given in the Appendix of the COPM booklet, in order to remain as neutral and congruent as possible; hence, the analysis could still be reproducible with the same results.

Lastly, our study was based on individuals' perceptions, which might be different from a real decrease in occupational participation. In France, for example, a study of 1771 chatbot users being followed up for breast cancer, asthma, depression, or migraine found that 38.06% suffered from psychological distress [34]. Another French study of 11,391 participants showed that women (77% of our sample), students (15% of our sample), disabled people, people with no access to outdoor spaces, and those living in a small home (44% of our respondents were living in a single- or two-level flat) were more at risk of having their wellbeing negatively impacted by the lockdown [35]. These characteristics might influence the perception of differences with the prepandemic period and the desire to engage in occupations.

Despite these limitations, our study provided in-depth qualitative and quantitative analyses of a large sample of occupations that were more frequently engaged in during lockdown. Our findings might be of great value in occupational science and might provide a better understanding of what the members of the general population choose to do when their usual occupations are disrupted.

### 4.7. Implications for Occupational Therapy Practice and Research

The global lockdown in the spring of 2020 led to various occupational transitions; many of the latter were not freely chosen. Given the link between occupational engagement and health, these changes might have had dramatic effects [36]. As stated by Hammell [8] “as occupational therapists, we have resources and knowledge […] to discover the occupations that can provide structure, routine and meaning within our disrupted lives.” A review of the functional impacts of the COVID-19 pandemic prepublished in May 2020 found that 32 studies had already investigated the impact of the pandemic on the general population [37].

Our results provided a better description of how different generations adjust to restrictions in their immediate environment. We notably found that when active leisure is disrupted, people of all generations maintained their occupational balance by reengaging in quiet leisure. We also found that younger generations were more inclined to engage in new occupations, while OAs preferred to engage more frequently in occupations they already knew.

Although occupational therapists usually know how to manage their clients' occupational disruptions, the global pandemic and its socioeconomic consequences may generate new challenges. The results presented here highlight the role that occupational therapists could take on by enabling occupational transitions during lockdown and helping people to manage disruptions in existing routines, such as working from home, job loss, and living in the same place all the time. As in other contexts of occupational disruption, occupational therapists have a range of solutions at their disposal: problem-solving has been found to be particularly helpful in the case of pandemics [38], as well as helping people to “take care of [themselves] and others, to experience a sense of belonging and connectedness, to foster a sense of self-worth, to experience pleasure, purpose and meaning through engagement in roles and occupations [they] value, to enact choices in our lives, and to experience hope and a sense of coherence and continuity within our lives” and thus reenabling occupational engagement [8]. Lastly, this period is generating unique opportunities for primary care provision with an occupational perspective. In fact, returning to previous occupations after a long period of disruption can be challenging for some people—especially those with cognitive and/or mental disorders. Occupational therapists can help these people return to their previous occupations, as illustrated by Mynard's guides on helping the general population to cope with lockdown [39] and the postlockdown situation [40].

## 5. Conclusions

Our results showed that lockdown led to (i) stronger engagement in quiet leisure by all generations of adults and (ii) new, satisfying forms of socialization—especially among older generations and despite the imposition of social distancing. Initially, one could have expected to see greater differences between generations. Furthermore, it would be worth investigating the independent associations between gender, the living environment, and some occupations in more detail. Spending more time at home also reduced generational differences in some occupations (e.g., cooking). These results help us to understand how human beings adapt to environmental restrictions to maintain some form of occupational balance. This information might help to understand how different generations engage in occupations after disruption. Occupational therapists may have a role in helping community-dwelling people to balance and structure their new daily routines.

## Figures and Tables

**Table 1:** Sociodemographic characteristics of the COPACO study's respondents.

	Total (*n* = 2534)	YAs	MAs	OAs	*p* value^∗^
Age					
Median (IQR)	41 (29-56)	28 (24-33)	49 (44-53)	68 (64-72)	<0.001
Range	(18-87)	(18-39)	(40-59)	(60-87)	
Sex, *N* = 2526					
Women	1941 (76.8)	960 (81.6)	633 (75.5)	348 (68.0)	<0.001
Place of living during lockdown, *N* = 2469					
Flat	1055 (42.7)	575 (49.2)	314 (38.3)	166 (34.7)	<0.001
House	1386 (56.1)	579 (49.5)	498 (60.7)	309 (64.5)	
Two-level flat	28 (1.1)	15 (1.3)	9 (1.1)	4 (0.8)	
Living environment during lockdown, *N* = 2520					
In an urban area or city	1659 (65.8)	779 (66.3)	556 (66.7)	324 (63.4)	0.4
People sharing the place of living during lockdown, *N* = 2533					
Same as usual	2490 (98.3)	1156 (98.1)	826 (98.5)	508 (98.5)	0.6
Usual professional status, *N* = 2531					
Student	372 (14.7)	350 (29.7)	22 (2.6)	0 (0.0)	<0.001
Part-time worker	277 (10.9)	105 (8.9)	150 (17.9)	22 (4.3)	
Full-time worker	1309 (51.7)	649 (55.1)	597 (71.4)	63 (12.2)	
Unemployed	79 (2.9)	41 (3.5)	27 (3.2)	5 (1.0)	
Retired	421 (16.6)	0 (0.0)	10 (1.2)	411 (79.7)	
Other	79 (3.1)	34 (2.9)	30 (3.6)	15 (2.9)	
Professional/study activity during lockdown, *N* = 2344					
Part-time homeworking/study	438 (18.7)	237 (20.3)	164 (19.9)	37 (10.5)	<0.001
Full-time homeworking/study	837 (35.7)	422 (36.1)	377 (45.8)	38 (10.8)	
Part-time at work/study place	196 (8.4)	116 (9.9)	69 (8.4)	11 (3.1)	
Full-time at work/study place	213 (9.1)	125 (10.7)	79 (9.6)	9 (2.6)	
No work/study	660 (28.2)	268 (23.0)	134 (16.3)	258 (73.1)	
Socioprofessional category, *N* = 1703					
Craftsman, trader, or company manager	97 (5.7)	39 (4.7)	47 (6.2)	11 (9.6)	<0.001
Employee	441 (25.9)	297 (36.0)	130 (17.1)	14 (12.2)	
Executive or intellectual professions	904 (53.1)	352 (42.6)	487 (63.9)	65 (56.5)	
Farmer	3 (0.2)	2 (0.2)	0 (0.0)	1 (0.9)	
Intermediate professions	236 (13.9)	123 (14.9)	91 (11.9)	22 (19.1)	
Worker	22 (1.3)	13 (1.6)	7 (0.9)	2 (1.7)	
Change of income during lockdown, *N* = 2429					
Total loss of income	112 (4.6)	70 (6.3)	33 (4.0)	9 (1.9)	<0.001
Major loss of income	130 (5.4)	77 (6.9)	45 (5.4)	8 (1.7)	
Partial loss of income	326 (13.4)	174 (15.6)	120 (14.4)	32 (6.7)	
No loss of income	1832 (75.4)	777 (69.4)	628 (75.6)	427 (89.1)	
Increase in income	29 (1.2)	21 (1.9)	5 (0.6)	3 (0.6)	

^∗^Pearson's chi-squared test or Student's *t*-test. YAs = younger adults; MAs = middle-aged; OAs = older adults; *n* (%), unless otherwise indicated.

**Table 2:** More frequently engaged occupations during lockdown in the COPACO study, by generation.

	Total (*n* = 4500) *n* (%)	Occupations more frequently performed by YAs (*n* = 2189), (48.6) *n* (%)	Occupations more frequently performed by MAs (*n* = 1456), (32.4) *n* (%)	Occupations more frequently performed by OAs (*n* = 855), (19.0) *n* (%)	*p* value^∗^	Pairwise comparison when the value for the domain or subdomain was <0.2; adjusted for the false discovery rate		
						YAs vs. MAs	YAs vs. OAs	MAs vs. OAs
*Leisure*	3016 (67.0)	1463 (66.8)	926 (63.6)	627 (73.3)	<0.001	0.04	0.002	<0.001

*Quiet recreation*	1717 (38.2)	851 (38.9)	485 (33.3)	381 (44.6)	<0.001	0.002	0.004	<0.001
Reading	424 (9.4)	193 (8.8)	120 (8.2)	111 (13.0)	<0.001	0.54	0.002	<0.001
Crafts	402 (8.9)	209 (9.6)	108 (7.4)	85 (9.9)	0.05	0.05	0.74	0.05
Needlework	171 (3.8)	71 (3.2)	49 (3.4)	51 (6.0)	0.001			
Drawing/painting	82 (1.8)	50 (2.3)	16 (1.1)	16 (1.9)	0.03			
Writing	32 (0.7)	12 (0.6)	10 (0.7)	10 (1.2)	0.2			
Creation of photo or video albums	22 (0.5)	13 (0.6)	5 (0.3)	4 (0.5)	0.6			
Crafts with children	14 (0.3)	7 (0.3)	7 (0.5)	0 (0.0)	0.1			
Other or not specified	81 (1.8)	56 (2.6)	21 (1.4)	4 (0.5)	<0.001			
Watching TV/series/movies	287 (6.4)	133 (6.1)	98 (6.7)	56 (6.6)	0.7			
Playing online/video games	118 (2.6)	96 (4.4)	17 (1.2)	5 (0.6)	<0.001	<0.001	<0.001	0.16
Playing board games	108 (2.4)	54 (2.5)	41 (2.8)	13 (1.5)	0.1	0.52	0.17	0.15
Listening/playing music	82 (1.8)	49 (2.2)	17 (1.2)	16 (1.9)	0.1	0.06	0.53	0.26
Using new technologies	69 (1.5)	16 (0.7)	17 (1.2)	36 (4.2)	<0.001	0.17	<0.001	<0.001
Playing individual intellectual games	54 (1.2)	24 (1.1)	13 (1.0)	17 (2.0)	0.1	0.55	0.09	0.09
Practicing meditation/relaxation	45 (1.0)	21 (1.0)	16 (1.1)	8 (0.9)	0.9			
“Keeping updated”	38 (0.8)	13 (0.6)	12 (0.8)	13 (1.5)	0.05	0.41	0.03	0.18
Going into the countryside	22 (0.5)	11 (0.5)	8 (0.6)	3 (0.4)	0.8			
Taking time to do things	20 (0.4)	7 (0.3)	9 (0.6)	4 (0.5)	0.4			
Sunbathing	15 (0.3)	9 (0.4)	3 (0.2)	3 (0.4)	0.6			
Taking photographs	5 (0.1)	4 (0.2)	0 (0.0)	1 (0.1)	0.2			
Attending online religious services	4 (0.1)	3 (0.1)	1 (0.1)	0 (0.0)	0.8			
Other or not specified	21 (0.5)	8 (0.4)	4 (0.3)	9 (1.1)	0.03	0.64	0.03	0.03
*Active recreation*	1101 (24.5)	534 (24.4)	364 (25.0)	203 (23.7)	0.8			
Participating in sports/physical activities	737 (16.4)	380 (17.4)	230 (15.8)	127 (14.9)	0.2			
Walking	132 (2.9)	38 (1.7)	54 (3.7)	40 (4.7)	<0.01			
Gym/fitness	113 (2.5)	51 (2.3)	39 (2.7)	23 (2.7)	0.8			
Yoga/pilates/qiqong	103 (2.3)	55 (2.5)	31 (2.1)	17 (2.0)	0.6			
Running	40 (0.9)	19 (0.9)	16 (1.1)	5 (0.6)	0.4			
Exercise bike	38 (0.8)	9 (0.4)	16 (1.1)	13 (1.5)	0.01			
Cycling	23 (0.5)	8 (0.4)	6 (0.4)	9 (1.1)	0.1			
Racket sports	10 (0.2)	5 (0.2)	4 (0.3)	1 (0.1)	0.8			
Dancing	10 (0.2)	6 (0.3)	2 (0.1)	2 (0.2)	0.7			
Other or not specified	268 (6.0)	189 (8.6)	62 (4.3)	17 (2.0)	<0.001			
Gardening	296 (6.6)	117 (5.3)	109 (7.5)	70 (8.2)	0.004	0.01	0.01	0.54
Playing with children	41 (0.9)	21 (1.0)	20 (1.4)	0 (0.0)	0.003	0.25	0.01	0.003
Caring for a pet	12 (0.3)	6 (0.3)	1 (0.1)	5 (0.6)	0.1	0.26	0.26	0.09
Other or not specified	1 (0.02)	1 (0.1)	0 (0.0)	0 (0.0)	1.0			
*Socialization*	198 (4.4)	78 (3.6)	77 (5.3)	43 (5.0)	0.03	0.03	0.09	0.79
Video calls with friends/family	82 (1.8)	39 (1.8)	28 (1.9)	15 (1.8)	0.9			
Talking on the phone	44 (1.0)	11 (0.5)	16 (1.1)	17 (2.0)	0.001	0.06	<0.001	0.08
Spending time with family	32 (0.7)	12 (0.6)	17 (1.2)	3 (0.4)	0.04	0.06	0.58	0.06
Using social media	23 (0.5)	8 (0.4)	12 (0.8)	3 (0.4)	0.2			
Other or not specified	17 (0.4)	8 (0.4)	4 (0.3)	5 (0.6)	0.5			

*Productivity*	1379 (30.6)	657 (30.0)	508 (34.9)	214 (25.0)	<0.001	0.003	0.01	<0.001

*Household management*	1082 (24.0)	500 (22.8)	402 (27.6)	180 (21.1)	<0.001	0.002	0.29	<0.001
Cooking	488 (10.8)	286 (13.1)	164 (11.3)	38 (4.4)	<0.001	0.11	<0.001	<0.001
Doing household chores	338 (7.5)	106 (4.8)	127 (8.7)	105 (12.3)	<0.001	<0.001	<0.001	0.006
Caring for children	125 (2.8)	56 (2.6)	62 (4.3)	7 (0.8)	<0.001	0.01	0.003	<0.001
DIY	119 (2.6)	46 (2.1)	45 (3.1)	28 (3.3)	0.1	0.09	0.09	0.81
Buying groceries	12 (0.3)	6 (0.3)	4 (0.3)	2 (0.2)	1.0			
*Paid/unpaid work*	151 (3.4)	65 (3.0)	72 (5.0)	14 (1.6)	<0.001	0.003	0.04	<0.001
Paid work	142 (3.2)	63 (2.9)	66 (4.5)	13 (1.5)	<0.001	0.01	0.03	<0.001
Unpaid work	8 (0.2)	2 (0.1)	5 (0.3)	1 (0.1)	0.2			
*Play/school*	146 (3.2)	92 (4.2)	34 (2.3)	20 (2.3)	0.002	0.01	0.02	1
Learning a foreign language	40 (0.9)	21 (1.0)	9 (0.6)	10 (1.2)	0.4			
Other or not specified	106 (2.4)	71 (3.2)	25 (1.7)	10 (1.2)	<0.001			

*Self-care*	105 (2.3)	69 (3.2)	22 (1.5)	14 (1.6)	0.002	0.01	0.03	0.81

*Personal care*	105 (2.3)	69 (3.2)	22 (1.5)	14 (1.6)	0.002	0.01	0.03	0.81
Resting	55 (1.2)	39 (1.8)	10 (0.7)	6 (0.7)	0.004	0.02	0.05	0.97
Personal appearance	24 (0.5)	16 (0.7)	6 (0.4)	2 (0.2)	0.2			
Feeding	13 (0.3)	8 (0.4)	4 (0.3)	1 (0.1)	0.6			
Healthcare	7 (0.2)	4 (0.2)	1 (0.1)	2 (0.2)	0.6			
Other or not specified	2 (0.04)	1 (0.1)	1 (0.1)	0 (0.0)	1.0			

^∗^Pearson's chi-squared test or Student's *t*-test. YAs = younger adults; MAs = middle-aged; OAs = older adults.

**(a):** 

	Leisure		Socialization		Quiet recreation		Productivity	
	OR (95% CI)	*p* value^∗^	OR (95% CI)	*p* value^∗^	OR (95% CI)	*p* value^∗^	OR (95% CI)	*p* value^∗^
Young adults	1.00		1.00		1.00		1.00	
Middle-aged adults	0.90 (0.65-1.24)	0.50	1.54 (1.02-2.32)	0.04	0.81 (0.64-1.02)	0.07	0.90 (0.71-1.13)	0.35
Older adults	0.99 (0.53-1.82)	0.95	1.37 (0.64-2.91)	0.42	0.64 (0.41-0.99)	0.05	0.82 (0.53-1.26)	0.36
Females	1.06 (0.74-1.52)	0.74	1.00 (0.63-1.57)	0.99	0.94 (0.72-1.23)	0.65	1.39 (1.07-1.80)	0.01
Place of living during lockdown (house vs. flat)	0.85 (0.61-1.19)	0.35	0.80 (0.53-1.22)	0.31	0.67 (0.52-0.85)	0.001	1.11 (0.88-1.41)	0.438
Living environment during lockdown (urban area vs. rural area)	0.90 (0.64-1.27)	0.54	1.27 (0.81-2.00)	0.30	1.15 (0.90-1.48)	0.26	1.09 (0.85-1.39)	0.49
Socioprofessional category								
Craftsman, trader, company manager, or farmer	1.00		1.00		1.00		1.00	
Executive or intellectual professions	1.01 (0.48-2.11)	0.99	0.66 (0.27-1.66)	0.38	0.88 (0.51-1.51)	0.64	0.93 (0.54-1.58)	0.78
Worker, employee, or intermediate professions	1.37 (0.65-2.90)	0.41	0.51 (0.20-1.30)	0.16	1.09 (0.63-1.86)	0.77	0.77 (0.45-1.31)	0.34
Change of income during lockdown								
Total or major loss of income	1.00		1.00		1.00		1.00	
Partial loss of income	1.03 (0.68-1.57)	0.88	0.67 (0.37-1.19)	0.17	1.00 (0.75-1.35)	0.98	1.07 (0.80-1.43)	0.66
No loss of income or increase in income	1.24 (0.70-2.18)	0.46	0.60 (0.28-1.29)	0.19	1.32 (0.90-1.95)	0.16	1.24 (0.85-1.81)	0.27
Country (France vs. other)	0.90 (0.56-1.44)	0.65	0.82 (0.47-1.42)	0.47	1.04 (0.75-1.44)	0.83	0.86 (0.62-1.18)	0.35

**(b):** 

	Household management		Play/school		Personal care		Paid/unpaid work	
	OR (95% CI)	*p* value^∗^	OR (95% CI)	*p* value^∗^	OR (95% CI)	*p* value^∗^	OR (95% CI)	*p* value^∗^
Young adults	1.00		1.00		1.00		1.00	
Middle-aged adults	0.94 (0.75-1.19)	0.63	0.87 (0.53-1.42)	0.58	0.71 (0.38-1.30)	0.26	1.22 (0.81-1.82)	0.34
Older adults	0.89 (0.57-1.38)	0.59	0.84 (0.32-2.20)	0.72	0.71 (0.21-2.39)	0.58	0.59 (0.23-1.54)	0.28
Female	1.54 (1.18-2.02)	0.002	0.81 (0.48-1.36)	0.42	0.97 (0.49-1.89)	0.92	0.89 (0.57-1.40)	0.63
Place of living during lockdown (house vs. flat)	1.11 (0.87-1.40)	0.41	0.54 (0.32-0.92)	0.02	0.43 (0.22-0.86)	0.02	1.26 (0.81-1.94)	0.30
Living environment during lockdown (urban area/city vs. rural area)	1.05 (0.82-1.34)	0.72	0.95 (0.56-1.61)	0.84	1.05 (0.54-2.06)	0.88	1.26 (0.81-1.94)	0.30
Socioprofessional category								
Craftsman, trader, company manager, or farmer	1.00		1.00		1.00		1.00	
Executive or intellectual professions	0.91 (0.54-1.54)	0.72	1.68 (0.58-4.85)	0.34	0.71 (0.18-2.88)	0.63	0.57 (0.27-1.20)	0.14
Worker, employee, or intermediate professions	0.85 (0.50-1.44)	0.55	2. 05 (0.72-5.84)	0.18	0.92 (0.23-3.67)	0.91	0.35 (0.16-0.75)	0.01
Change of income during lockdown								
Total or major loss of income	1.00		1.00		1.00		1.00	
Partial loss of income	1.07 (0.80-1.44)	0.64	1.62 (0.91-2.88)	0.10	0.79 (0.36-1.73)	0.55	0.69 (0.38-1.26)	0.22
No loss of income or increase in income	0.89 (0.61-1.30)	0.55	3.18 (1.73-5.86)	<0.001	0.78 (0.29-2.13)	0.63	1.36 (0.74-2.50)	0.33
Country (France vs. other)	1.13 (0.81-1.56)	0.48	0.76 (0.42-1.39)	0.38	1.09 (0.47-2.49)	0.84	0.56 (0.34-0.93)	0.03

^∗^Wald's test. OR (95% CI): adjusted odds ratio (95% confidence interval) in a multivariate logistic regression. All variables were adjusted for sex, place of living during lockdown, living environment during lockdown, socioprofessional class, change of income during lockdown, and country of residence.

**Table 4:** Participants' ratings of leisure occupations in the COPACO study.

	YAs median (IQR)	MAs median (IQR)	OAs median (IQR)	*p* value
Importance	8 (6; 9)	8 (6; 10)	8 (7; 10)	<0.001
Performance (difference in the score on a 1-to-10 scale for lockdown vs. prepandemic)	+5 (3; 6)	+4 (3; 6)	+3 (1; 5)	<0.001
Satisfaction (difference in the score on a 1-to-10 scale for lockdown vs. prepandemic)	+3 (0; 5)	+3 (0; 5)	+2 (0; 4)	<0.001

YAs = younger adults; MAs = middle-aged; OAs = older adults.

**Table 5:** Participants' ratings of productivity in the COPACO study.

	YAs median (IQR)	MAs median (IQR)	OAs median (IQR)	*p*
Importance	8 (7; 10)	8 (7; 10)	8 (7; 9)	<0.01
Performance (difference in the score on a 1-to-10 scale for lockdown vs. prepandemic)	+4 (2; 5)	+3 (2; 5)	+3 (2; 5)	0.07
Satisfaction (difference in the score on a 1-to-10 scale for lockdown vs. prepandemic)	+3 (0; 5)	+2 (0; 4)	+2 (0; 4)	0.0006

YAs = younger adults; MAs = middle-aged; OAs = older adults.

**Table 6:** Participants' ratings of self-care occupations in the COPACO study.

	YAs median (IQR)	MAs median (IQR)	OAs median (IQR)	*p* value
Importance	8 (7; 10)	8 (7; 10)	9 (8; 10)	0.6
Performance (difference in the score on a 1-to-10 scale for lockdown vs. prepandemic)	+4 (3; 6)	+4.5 (3; 6)	+1 (3.5; 6)	0.5
Satisfaction (difference in the score on a 1-to-10 scale for lockdown vs. prepandemic)	+3 (1; 6)	+5 (0; 6)	+2 (0; 4)	0.5

YAs = younger adults; MAs = middle-aged; OAs = older adults.

## Data Availability

The data used to support the findings of this study are available from the corresponding author upon request.
